# The Lower Limb Movements of the Fetus in Uterus: A Narrative Review

**DOI:** 10.1155/2023/4324889

**Published:** 2023-01-23

**Authors:** Xiaoxue Zhao, Jan Awrejcewicz, Jianpeng Li, Yuhuan He, Yaodong Gu

**Affiliations:** ^1^Faculty of Sports Science, Ningbo University, Ningbo, China; ^2^Department of Automation, Biomechanics and Mechatronics, Lodz University of Technology, Lodz, Poland; ^3^Department of Physical and Health Education, Udon Thani Rajabhat University, Udon Thani, Thailand

## Abstract

The fetus movements play an important role in fetal well-being. With the continuous advancement of real-time scanning machines, it is feasible to observe the fetus movement in detail. The characteristics of fetal lower limb movements in prenatal examination have not been systematically investigated. This review proposes the patterns of fetal lower limb movements, the maternal influence on fetal lower limb movements, and the application of fetal lower limb movements for the diagnosis of prenatal diseases. A systematic search of literature on the lower limb movements of the fetus in uterus was performed in the databases, namely, Web of Science and Scopus. Thirty-four publications were selected. This review demonstrates that isolated fetal lower limb movements are rare and always accompanied with the movements of other body segments. Detection of the presence of fetal leg movements seems to be of no diagnostic value for fetuses with prenatal diseases. The isolated lower limb movement was statistically significant different between fetuses of low- and high-risk pregnant women. The coordinated movements of the fetal lower limbs and other parts should be considered when analyzing fetal movements in the future study.

## 1. Introduction

Fetus movement has long been a subject of extreme importance in the fetal growth and development. The detection and description of fetus movements offer important information on the development of intrauterine and fetal well-being [1]. Consequently, the observation and record of fetal movements by real-time scanning machines in uterus have been universally performed to evaluate the fetal well-being [2–4]. With the emergence of modern real-time scanning equipment, more accurate and detailed visualization and monitoring of fetal movement become possible. The first fetal movement occurred during the 7th week of pregnancy observed by the real-time scanning machine [5]. The isolated leg movements first appeared between 9 and 12 weeks [6]. Different specific fetal movement patterns and their occurrence were identified and clarified [7, 8]. Fetal movements in uterus involving lower limb include isolated leg movements [6, 9–11], body rotation [5], startle [7, 12], general movements [6], stretching [9], kicking [5], and jumping [11].

The spontaneous movement is an expression and reflection of early neural activity, knowledge of normal development of fetus movements, and the assessment of the quality of fetus movement that might shed light on the integrity of the nervous system and neural development [6, 13]. Thus, the examinations of spontaneous leg movements are applied to determine the segmental level of neural tube lesion [14]. In the past, the absence or presence of fetal leg movements was used to diagnose the neural tube defects of the fetus [15]. Defects of early neonatal motor ability could indicate the effect of postnatal gravity on preexisting neurodevelopmental abnormalities [16]. The absence of lower limb movements may be as a contraindication to fetal myelomeningocele repair [17]. Fetal prenatal surgery should be launched in fetuses without lower limb movements in early gestation to keep the movement ability of legs [18]. This study has shown that compared to postnatal repair of myelomeningocele, prenatal surgery for myelomeningocele improved the independent-walking rate [19].

The fetal lower limb movements are essential for the examination of fetal neural development, but the characteristics of fetal lower limb movements have not been systematically investigated. This review proposes the patterns of fetal lower limb movements, the maternal influence on fetal lower limb movements, and the application of fetal lower limb movements for the diagnosis of prenatal diseases.

## 2. Materials and Methods

### 2.1. Focused Question Based

The focused question was selected by the Preferred Reporting Items for Systematic Reviews and Meta-Analyses 2020 guidelines. The focus was on the lower limb movements of the fetus in uterus.

### 2.2. Eligibility Criteria

The following eligibility criteria were required: (1) only studies included the fetal lower limb movements; (2) studies concerned human fetus in uterus; and (3) published articles were written in English language and do not include historical reviews, book chapters, encyclopedia, correspondence, and short communications.

### 2.3. Search Strategy and Study Selection

The literature search was performed in the following databases: Web of Science and Scopus. All publications from 1965 up to May 2022 were included in this literature search. The literature search terms were the following combination of keyword string: “fetus” and “lower extremity movement” or “lower limb movement” or “leg movement.” Two different authors examined and checked the titles and abstracts of studies for consistency according to the stated eligibility criteria. Structured algorithm was used to select and check the articles (Figure 1).

## 3. Results

### 3.1. The Lower Limb Movements of the Fetus in Uterus

Frequencies of lower limb movements have increased significantly from 12 to 19 weeks in singleton fetuses in comparison with twin fetuses [20]. Fetal leg movements were synchronized and harmonized with fetal head, mouth, arm, and trunk movements [21]. Fetal lower limb movements were frequently presented before the gestation of 28 weeks and after 28 weeks, the rate was decreased [22]. Additionally, this work highlighted that the occurrence of lower limb movements was extremely high and even same as the incidence of the arm movements. The occurrence of leg movements in fetuses above 30 weeks was significantly decreased in contrast to fetuses at 18–25 weeks [23]. The leg movements were mainly involved with the hip rotation. From 30 to 37 weeks, the number of lower limb movements in 1 min declined, and number of leg movements by minute of male fetuses was greater than female fetuses [24].

#### 3.1.1. Isolated Leg Movements

The isolated leg movements first appeared between 9 and 12 weeks [6]. It is difficult to observe fetal leg movements alone, and there is no developmental trend in isolated leg movements. The rapid and jerky lower limb movements can occur as single movements (twitches) or in rhythmic movements (clonus) about three to four times per second. Leg clonus can be seen only after 14 weeks, but it is also rare. A further longitudinal study included 12 fetuses in the first half of pregnancy revealed that isolated leg movements were not frequently occurring and did not show developmental trends [7]. Lu et al. [9] studied 50 fetuses using real-time 3D ultrasound for 10 min to observe the fetal movements; they found that the frequency and incidence of isolated lower limb movements were lower than general movements and startle. The isolated leg movement was secondary to the arm movements at 17–19 weeks [25]. In addition, there was no statistical significance in the number of isolated lower limb movements between 14–16 and 17–19 weeks. Although these studies have shown that the sole movement of the fetal legs has been observed, some studies have even used the sole movement of the fetal legs as a reference index for the diagnosis of fetal prenatal diseases; other studies stated that the fetal lower limb movements are combined with the movements of other parts of the fetus [21, 22].

#### 3.1.2. Fetal Body Rotation

Fetal body rotation refers to the fetus rolls from side to side; this movement was very active with all parts of its body involved, and the legs kicked the gestational sac wall with the flexion and extension of the feet [5]. Fetal body rotation often concerns with the change of lower limb movements and could be observed near the sagittal or transverse axis [6]. Rotation of the fetus might result from leg movements with hip rotation or head rotation accompanied by trunk rotation or even the combination of the three rotation movements. AboEllail et al. [20] observed that both singleton and twin fetuses had an average of three body rotations within 15 min at 12–13 weeks. The difference of body rotation of fetuses between 14–16 and 17–19 weeks was not significant [25]. The frequency of body rotation in twin fetuses was decreased from 12 to 19 weeks [20].

#### 3.1.3. General Movements

General movements were typically defined as a series of variable speed and amplitude motions, and lasted from a few seconds to around 1 min [9]. Same as for fetal body rotation, all parts of the body participated in this movement, but without distinctive pattern. The majority of arms and legs extended and flexed with superimposed rotation, and often the direction of the movement slightly changed. This movement had the highest incidence of 100% present during 10 min real-time three-dimensional ultrasound observation at 11–14 weeks [9]. General movements rate generally raised from 8 to 10 weeks and reached a plateau at 10 weeks; the longest interval between general movements was longer than the longest duration of fetal inactivity observed in 12 fetuses of different gestations [7]. For twin fetuses at the gestation of 12–13 weeks, the frequency of general movements was significantly larger than that of other fetal movements [20]. At the gestation of 12–19 weeks, the rate of occurrence of general movements significantly decreased in both singleton and twin fetuses [26].

#### 3.1.4. Startle

The startle is characterized by the flexion or extension of the limbs and first appeared at 8–9 weeks [6]. The fetal limbs are usually greatly flexed or extended, but sometimes the amplitude is small or even imperceptible. Startles tended to increase in 8–9 weeks, but gradually decreased from 9 weeks and often recurred at about 10 s intervals during the first half of gestation [7]. Startle was regularly detected as a single movement [22].

#### 3.1.5. Kick

Fetus kicks against the uterine wall which was commonly of strong strength, followed by slowly return into its original position [5]. Fetal step, similar to a kick, showed vigorous limb movements and always accompanied with the whole trunk movements in the second half of gestation [22]. Jumping movements were one of the most frequent fetal movements at 12–13 weeks and its frequency significantly raised from 10–11 to 12–13 weeks [10]. Stroking-like movements occurred around 18 weeks of gestation, and kicking occurred irregularly at all gestations [23]. In addition, the quantitative analysis of the kicking movement and plantar flexion action of the fetuses at different gestational ages also suggested that the knee range of motion decreased with progressive gestational weeks [27]. Furthermore, this study which investigated the joint angular velocity of fetuses demonstrated that the mean knee joint angular velocity of fetuses at 30 weeks was significantly higher than that at 24 weeks, and the kick force significantly elevated from 20 to 30 weeks [28]. The average reaction force when kick against the uterus wall calculated by computational finite element simulation was 0.52 ± 0.15 N at 20–22 weeks [29].

### 3.2. Maternal Influence on Fetal Lower Limb Movement

The Kurjak antenatal neurodevelopmental test (KANET) for fetal neurobehavior was introduced for prenatal assessment by the use of three-dimensional or four-dimensional sonography [30]. In this prenatal assessment, the characteristics and significance of normal and abnormal fetal isolated leg movements and general movements were investigated. The difference of isolated lower limb movement between fetuses of low- and high-risk pregnant women investigated by KANET was statistically significant [31]. There were statistical significant differences of isolated leg movements between low- and high-risk pregnant women during 2nd and 3rd trimesters [3]. Through 1-year longitudinal cohort study of the isolated leg movements in KANET, there was significant difference in individual KANET parameters between the fetuses of low- and high-risk pregnant women [2]. Miskovic et al. [4] compared the isolated leg movements between 116 high-risk pregnant women and 110 pregnant women by using the modified KANET. The character of fetal lower limb movements and general movements was classified into three levels. The difference of isolated leg movement between high- and low-risk pregnant women was not statistically significant, while statistical significance was shown for general movements. Hanaoka et al. [32] evaluated the maternal ethnic influences in fetal behaviors between Asian (89 Japanese) and Caucasian pregnant women (78 Croatian) at 28–38 weeks by using the KANET. Significant differences were noted in isolated movements, while no statistical significance was found in gestalt of general movements between Asian and Caucasian pregnant women. Habek [10] studied on the impact of maternal smoking in early pregnancy on fetal movements by using transvaginal two-dimensional sonography for 5 min; no significant difference was observed in isolated spontaneous lower limb movements with nonsmoking pregnant women, and pregnant women daily intake an average of 10 or 20 cigarettes. Bartha et al. [33] investigated the influence of maternal anxiety on fetal behaviors (startle, general movement, isolated leg movement, and stretch) at 15 weeks' gestation; they observed that maternal glucose was significantly associated with isolated leg movements and startles. Amniotic fluid catecholamines were significantly correlated with movement involving legs (startles and general movements).

### 3.3. Diagnosis of Prenatal Diseases by Fetal Lower Limb Movements

#### 3.3.1. Prenatal Diagnosis of Spina Bifida Aperta by Fetal Lower Limb Movement

For fetuses with spina bifida aperta, leg movements caudal to the meningomyelocele are often observed; however, the movement disappeared shortly after delivery. It remains to be seen that the absence of leg movements is the result of the neurodevelopmental malformation or superposed traumatic damage [34]. Parra et al. [12] studied 29 spinal muscular atrophy carrier couples who had at least one previous child with severe spinal muscular atrophy. All fetuses presented isolated lower limb movements in this study. The observation of the leg movements caudal to the meningomyelocele in six fetal spina bifida aperta at 16–40 weeks by using ultrasound demonstrated that fetal leg movements persistently presented. However, in two fetuses, the quality of leg movements caudal to the myelomeningocele was difficult to discern [34]. Verbeek et al. [35] studied six spina bifida aperta at an average of 34 weeks and 11 controls at an average of 28 weeks; they stated that despite the presence of fetal leg movements caudal to the meningomyelocele, muscle ultrasound density was greater than in age-matched controls and did not increase with advancing gestation. However, muscle ultrasound density was increased with advancing gestation in healthy fetus [35] and children [36].

#### 3.3.2. Prenatal Diagnosis of MMC by Fetal Lower Limb Movement

Carreras et al. [37] illustrated that the presence and absence and patterns of leg movements in sagittal planes provided a more reliable prognosis about the walking ability after birth compared to the anatomical level of lesion. Furthermore, Maroto et al. [38] elucidated this ultrasonographic finding and assessed the fetal lower limbs in the sagittal plane in 28 fetuses with myelomeningocele at 20.6–24.5 weeks. It has been found that the characteristics of the fetal ankle movements were described by the arch amplitude and the arch should be >45°. Farmer et al. [18] measured the presence of lower limb movements (the ankle, knee, and hip joint) in 183 fetuses with myelomeningocele by using ultrasound; the presence of these movements at baseline was significantly correlated with independent ambulation at 30 months for patients undergoing prenatal surgery. All 39 of those with walking ability after birth had hip movements and 38 had knee movements. Nine patients received prenatal surgery and could not walk; they did not have hip movement at baseline, and none of those could walk independently after birth. The fetal lower limb movement increased between postoperative days 1 and 5 after open fetal meningomyelocele repair; fetal knee and hip movements observed by using ultrasound at 32 weeks were correlated with ambulation at 30–36 months [39].

#### 3.3.3. Prenatal Diagnosis of Other Congenital Diseases by Fetal Lower Limb Movement

Warsof et al. [40] assessed the fetal leg movements and urologic systems in 120 fetuses with either neural tube defects or intracranial malformations. The results shown that fetal lower limb movements were persistly presented in most of the affected fetuses; it seems that the presence of fetal lower limb movements and the integrity of urinary tract seem to do not have diagnostic value. Another study of fetuses of 29 spinal muscular atrophy carrier couples at 11–14 weeks by using two-dimensional transabdominal ultrasound demonstrated that isolated lower limb movements were presented in all of them, while general movements and startle were observed in large majority of cases [12]. Weak leg movements were observed in a fetus diagnosed with diastematomyelia at 21 weeks by using dynamic-balanced-fast-filled-echo sequences cine MRI [41]. Another case study of a fetus with Déjerine–Sottas syndrome at 33 weeks found that the involvement, amplitude, and speed of the general movements and isolated leg movement were reduced [42]. Systematic assessment of fetal lower limb-related movements for 2 weeks has additional value to distinguish arthrogryposis multiplex congenita, fetal akinesia deformation sequence, and bilateral pes equinovarus [43]. More specifically no matter what the gestational age, the high-risk population of fetal akinesia deformation sequence presented abnormal quality in all fetuses within 2 weeks.

## 4. Conclusion

In summary, this review demonstrates that isolated fetal lower limb movements are rare and always accompanied with the movements of other parts of the fetus. There was a statistical significance for isolated leg movement between fetuses of low- and high-risk pregnant women. The absence or presence of isolated fetal lower limb movements does not have diagnostic value in fetuses with neural tube defects or other central nervous system malformations. The coordinated movements of the fetal lower limbs and other parts should be considered when analyzing fetal movements in the future study.

## Figures and Tables

**Figure 1:** Flowchart of the literature search.

## Data Availability

All data are included within this article.
